# PLK4 Is a Potential Biomarker for Abnormal Tumor Proliferation, Immune Infiltration, and Prognosis in ccRCC

**DOI:** 10.1155/2022/6302234

**Published:** 2022-09-20

**Authors:** Chenglu Hu, Qingping Liu, Chengyi Hu, Ying Wang, Pan Wang, Xing Zhou

**Affiliations:** ^1^School of Pharmacy and Bioengineering, Chongqing University of Technology, Chongqing 400054, China; ^2^Department of Pharmacy, Chongqing Hospital of Traditional Chinese Medicine, Chongqing 400011, China; ^3^Chongqing Key Laboratory of Medicinal Chemistry & Molecular Pharmacology, Chongqing University of Technology, Chongqing 400054, China

## Abstract

**Background:**

PLK4 is highly expressed and associated with poor prognosis in various malignancies. However, the role of PLK4 in clear cell renal cell carcinoma (ccRCC) is still unclear. This study is aimed at analyzing the expression, the potential regulating mechanism, and the role of PLK4 in the ccRCC by bioinformatics.

**Methods:**

PLK4 mRNA expression data and methylation levels in ccRCC were examined using TIMER, UALCAN, MethSurv, NCBI-GEO, and UCSC databases. Quantitative real-time PCR verifies the regulatory relationship between PLK4 and has-miR-214-3p. The GEPIA2 and STRING databases were used to find similar genes of PLK4 and then enriched with *R* language to analyze their similar genes. Correlations between PLK4 and tumor-infiltrating immune cells and cytokines exerting immunosuppression were analyzed using the TIMER database and the TISIDB databases.

**Results:**

PLK4 mRNA expression levels were significantly higher in ccRCC tissues than in paracancerous tissues. ccRCC tissues had lower DNA methylation levels of PLK4 than normal tissues. Importantly, the high PLK4 expression was associated with poor prognosis in ccRCC patients. The has-miR-214-3p negatively regulates the expression of PLK4. GO and KEGG pathway analysis showed that PLK4 coexpressed genes were mainly associated with multiple immune-related pathways, including cytokinesis, sister chromatid adhesions, and mitotic nuclear division. Our data suggest that the PLK4 expression is closely related to the level of immune infiltration and the cytokines that exert immune suppression, and IPS was significantly higher in the PLK4 low expression group.

**Conclusion:**

The PLK4 expression is associated with the prognosis of ccRCC patients and affects the immune microenvironment of ccRCC, and PLK4 is expected to be a new target for the diagnosis and treatment of ccRCC.

## 1. Introduction

Renal cell carcinoma (RCC), a tumor of the genitourinary system, is one of the common malignant tumors [1, 2]. Among the histological subtypes of renal cell carcinoma, clear cell renal cell carcinoma (ccRCC) is the most common subtype, accounting for 75% of all renal tumors. It has been proved that advanced patients bearing ccRCC have a poor prognosis and low survival [2, 3]. The main reasons for the poor prognosis include the limited effectiveness of chemotherapy and radiotherapy treatment [4, 5]. Although the rapid development of targeted therapy and immunotherapies brings new hope to the treatment of ccRCC, these therapies still do not achieve optimal therapeutic results in ccRCC, due to the limited available molecular targets (tyrosine kinase and mTOR signaling pathways), drug resistance, immune suppression, and tumor heterogeneity [6–9]. As a highly immune-infiltrated tumor [10], the proliferation of the tumor cells and the immune suppression provided by the tumor microenvironment are two keys in the process of tumorigenesis and progression [11]; thus, it is important to search for key biomarkers regulating both of tumor cell proliferation and tumor immune microenvironment, to establish a potential effective treatment option.

The centrosome is an important organelle, the center of microtubule organization in animal cells and some plant cells, which is closely related to processes such as mitosis and regulates cell cycle progression [12]. The number of centrosomes is regulated by centrosome replication factors [13], and an abnormal number of centrosomes lead to an abnormal chromosome state, which is closely related to tumorigenesis and development [14]. PLK4 is a serine/threonine-protein kinase with a C-terminal polo-box catalytic structural domain [15], which can regulate centriole replication through its phosphorylation [16], but the abnormal expression of it would lead to genomic instability and tumorigenesis via an abnormal upregulation of centrosome number [17]. Thus, as an important regulator of cell division, PLK4 plays an important role in the process of tumorigenesis and development [18]. Many studies have shown that PLK4 is expressed at abnormal levels in various cancer types, but different levels in different cancer types. However, the expression of PLK4 compared to paracancerous tissue in different tumor types is different. For example, PLK4 is highly expressed in breast cancer but low in hepatocellular carcinoma [19, 20]. Therefore, the role of PLK4 is equally controversial. Some studies have shown that the high PLK4 expression is positively correlated with low survival rates for lung cancer and can promote the invasion and metastasis of cancer [21, 22]. In contrast, in hepatocellular carcinoma, PLK4 was considered as a inhibitory factor of tumorigenesis and progression [20]. Obviously, PLK4 plays an important and tumor heterogeneous role in tumorigenesis and development, while its expression and role in ccRCC have not been revealed.

To reveal the expression and role of PLK4 in ccRCC, we performed a comprehensive analysis of PLK4 in ccRCC by bioinformatics using multiple available databases. We explored the expression and prognostic value of PLK4 in ccRCC and miRNAs acting on PLK4 followed by DNA methylation analysis. GO and KEGG analyses were then performed. Next, the correlation of the PLK4 expression in ccRCC with immune cells and immunosuppressive cytokines that make up the immune microenvironment of the tumor was analyzed. In conclusion, our study suggests that PLK4 may be a potential biomarker for aberrant tumor proliferation and immune infiltration and prognostic relevance in ccRCC and may also be a new immune-related therapeutic target.

## 2. Methods

### 2.1. Analysis of PLK4 Differential Expression

The Tumor Immunity Assessment Resource (TIMER) website (https://cistrome.shinyapps.io/TIMER/) is a comprehensive resource for the molecular characterization of tumor-immune interactions [23]. To assess the difference in the PLK4 expression between tumor and normal tissues adjacent to cancer, this study investigated the mRNA expression of different cancer types in TCGA (The Cancer Genome Atlas) using the TIMER database.

UALCAN (http://ualcan.path.uab.edu/index.html) is a website for online analysis of cancer genetic data, mainly based on relevant cancer data from the TCGA database [24]. To evaluate the difference in the PLK4 expression in tumor and paraneoplastic tissues, RNA sequence data from ccRCC were studied using the UALCAN database, and the mRNA expression levels of PLK4 between primary tumor and paraneoplastic tissues were analyzed.

The Gene Expression Omnibus (GEO) database (https://www.ncbi.nlm.nih.gov/geo/) is built and maintained by the National Center for Biotechnology Information (NCBI) [25]. It contains gene expression data submitted by research institutions around the world, mainly including gene chips and high-throughput sequencing data. Renal clear cell carcinoma data were downloaded from the NCBI-GEO database, dataset GSE53757, which included 72 normal samples and 72 tumor samples. Data were analyzed and plotted using the *R* packages limma, ggplot2, and ggpubr.

The UCSC database (https://genome.ucsc.edu) provides high-quality visualization of genomic data and genome annotation [26]. The expression profile data of ccRCC, including 72 paracancerous tissues and 535 tumor tissues, were downloaded from the UCSC database to screen paired sample information, with a total of 72 tumor samples and corresponding 72 paracancerous samples, and data analysis and mapping were performed using the *R* packages limma, ggplot2, and ggpubr.

The GEPIA2 website (http://gepia2.cancer-pku.cn/#index) database is one of the preferred tools for exploring large cancer genomic data and is a resource for processing TCGA data for differential gene expression, correlation, survival prognosis, etc. [27] To analyze the expression of PLK4 in various cancer stages, the expression of PLK4 in different pathological stages of various cancers can be obtained by analysis using the GEPIA2 database.

### 2.2. Micro-RNA Expression Analysis and Quantitative Real-Time PCR

ENCORI (https://starbase.sysu.edu.cn/) [28], TargetScan (https://www.targetscan.org/vert_80/) [29], and TANRIC (https://ibl.mdanderson.org/tanric/_design/basic/main.html) [30], the three databases, are web resources for predicting the interaction between target genes and miRNAs. The miRNAs acting on PLK4 were predicted using these three databases, then the intersection of the miRNAs obtained from the three databases was obtained using Veen plots, and the resulting miRNAs were observed in the ENCORI database for their differential expression in ccRCC and cancerous tissues.

The human ccRCC cell line ACHN was purchased from the Chinese Academy of Sciences, Shanghai Institutes for Biological Sciences (Shanghai, China). Cells were cultured in a 37°C incubator containing 5% CO_2_. ACHN cells were trypsinized when the cell fusion rate reached 80% and suspended in the culture medium. The cell suspension was inoculated into 12-well plates at a density of 2 × 10^5^ cells/mL. The has-miR-214-3p mimics (sense 5′-UUCUCCGAACGUGUCACGUTT-3′; antisense 5′-ACGUGACACGUUCGGAGAATT-3′) were purchased from Gema (Shanghai, China). The experiments were grouped into the microRNA NC group and microRNA mimic group. Total RNA samples were isolated using TRIzol (TIANGEN, China). RNA concentration was measured by NanoDrop One (Thermo Fisher, USA). cDNA was synthesized using a reverse transcription kit (Vazyme, China). Premix for qPCR reactions was prepared (Vazyme, China), and then qPCR reactions were performed on a fluorescent quantitative PCR machine (LightCycler 96, USA). The relative mRNA levels were normalized to the level of GAPDH and calculated using the 2^-*ΔΔ*Ct^ algorithm. The primers were manufactured by DynaBio (Chongqing, China). The primer sequences are as follows. PLK4, forward: GACACCTCAGACTGAAACCGTAC, reverse: GTCCTTCTGCAAATCTGGATGGC; GAPDH, forward: AATGGGCAGCCGTTAGGAAA, reverse: GCGCCCAATACGACCAAATC.

### 2.3. Survival Prognosis Analysis

The Kaplan-Meier plotter website (http://kmplot.com/analysis/index.php?p=background) was able to assess the effect of the PLK4 gene on survival in most cancers [31]. We used Kaplan-Meier Plotter and performed a survival analysis of PLK4 to plot survival curves of the effect of high and low expression levels of PLK4 on the OS stage of ccRCC in the database.

### 2.4. DNA Methylation of PLK4 and Its Prognostic Value in ccRCC

DNA methylation status is significantly correlated with gene expression levels and affects the prognosis of cancer patients [32]. To further determine the mechanism of PLK4 expression level upregulation in ccRCC, the PLK4 gene was entered into the TCGA platform of the UALCAN web, and tumor type and “methylation” were selected in the related module to obtain the methylation level of the PLK4 gene between tumor tissue and paracancerous tissue in ccRCC. In addition, we also analyzed the methylation levels of different pathological stages and tumor stages.

The cBioPortal contains DNA methylation levels [33],

First of all, we logged into the cBiPortal web (http://www.cbioportal.org/) to download the ccRCC methylation data. Then, the RNA expression data of ccRCC were downloaded from the UCSC website, and finally, the correlation analysis of PLK4 methylation with its expression was performed in the *R* language. We further used MethSurv web (https://biit.cs.ut.ee/methsurv/) to analyze the DNA methylation site information and degree of methylation of PLK4 in ccRCC and the prognostic value of these CpG sites.

### 2.5. GO and KEGG Pathway Enrichment Analysis of PLK4-Related Gene

STRING website (https://string-db.org/) is an online database for querying interactions between known proteins and predicting protein interactions [34]. To search for genes differentially expressed with PLK4, we first logged into the STRING website, entered "PLK4” in the “ Single Protein by Name/Identifier” module. We searched for “auto-detect/Homo sapiens.” Then, we set the following main parameters: in the “meaning of network edges” panel, we selected “evidence,” in the “active interaction sources” panel, and “experiments” in the “minimum required interaction score “ panel, selecting “medium confidence (0.400)”, and select “max number of interactors to show” panel Select “no more than 50 interactors” in the “1st shell” section. Finally, 17 binding proteins of PLK4 were obtained for the available experimental assays. We used the “Similar Gene Detection” module of GEPIA2 to obtain the top 50 PLK4-related target genes based on the dataset of ccRCC in all TCGAs. In addition, we also applied the “Gene_Corr” module of TIMER2 to analyze the top five highly correlated genes of PLK4, including the purity-adjusted Spearman's rank correlation test for partial correlation (cor) and *p* value. We combined the two sets of data and left 64 genes after deleting duplicates, and the screened genes were subjected to KEGG (Kyoto Encyclopedia of Genes and Genomes) pathway analysis and GO (Gene Ontology) enrichment analysis using the *R* package clusterProfiler [35], respectively.

### 2.6. Immune Infiltration Analysis

To investigate the relationship between PLK4 expression and immune cells, the TIMER database was used to determine the relationship between RNA sequence expression profile data of PLK4 in ccRCC and immune cells. The TIMER, CIBERSORT, CIBERSORT-ABS, TIDE, QUANTISEQ, XCELL, MCPCOUNTER, and EPIC algorithms were applied for immune infiltration estimations. Immune cells include cancer-associated fibroblast, neutrophils, myeloid dendritic cells, active CD4^+^ T cells, CD8^+^ T cells, endothelial cells, monocytes, macrophage M1, macrophage M2, and NK cells. We explored these genetic markers from those cited in previous publications [36–38].

TISIDB web (http://cis.hku.hk/TISIDB) contains a large amount of tumor immune-related data to analyze the relationship between gene expression and the immune system in individual tumors and to help predict immune therapy response [39]. We analyzed the relationship between PLK4 expression and immunosuppression in the TISIDB web. “rho” values greater than 0.2 and less than -0.2 and *p* < 0.05 were considered to be significantly correlated. The cytokines that exerted immunosuppression that was positively and strongly correlated with the PLK4 expression were then selected, and their correlation in ccRCC was plotted in scatterplots.

### 2.7. Correlation between PLK4 and Immunophenoscore (IPS) Analysis

The Cancer Imaging Archive (TCIA) database (http://tcia.at) collects a rich dataset of tumor images, and to assess the impact of high and low PLK4 expression on the effectiveness of immunotherapy in patients, we obtained IPS-related data from the TCIA database; we classified patients into those with low and high PLK4 expression. The IPS calculation process was performed as described in this article [40]. The higher the score, the better the immune checkpoint treatment effect.

### 2.8. Statistical Analysis

Online analysis was performed using the database default statistics. Differences in the PLK4 expression in cancerous and paraneoplastic tissues were performed by *t*-test. Kaplan-Meier was used for PLK4 survival analysis by log-rank test. *p* value of 0.05 was considered statistically significant.

## 3. Results

### 3.1. PLK4 Is Upregulated in ccRCC

According to the results obtained from the TIMER database, the PLK4 expression was significantly higher in uroepithelial carcinoma of the bladder, invasive breast cancer, squamous, and adenocarcinoma of the cervix, bile duct cancer, colon cancer, esophageal cancer, squamous cell carcinoma of the head and neck, renal suspicious cell carcinoma, renal clear cell carcinoma, renal papillary cell carcinoma, gastric cancer, thyroid cancer, and endometrial cancer, than in normal tissue (Figure 1(a)). To further determine the expression of PLK4 in ccRCC, we separately analyzed the gene expression levels of PLK4 between renal clear cell carcinoma and its paraneoplastic tissues using the UALCAN database, and PLK4 was highly expressed in renal clear cell carcinoma tissues compared to normal tissues (Figure 1(b)).

To further verify the reliability of differential gene expression, we downloaded the dataset GSE53757 of renal clear cell carcinoma from the GEO database and analyzed the differential expression of PLK4 in normal and cancer tissues by *R* language, and the results showed that PLK4 was highly expressed in cancer tissues compared with normal tissues (Figure 1(c)).

Meanwhile, we screened the expression profiles of renal clear cell carcinoma and its corresponding paired paraneoplastic tissues included in the TCGA database, followed by the analysis of the differential expression of PLK4 in tumor and its corresponding paired paraneoplastic tissues by *R* language, and the results showed that PLK4 was highly expressed in tumor tissues compared with paracancerous tissues (Figure 1(d)). We continued our in-depth study according to different pathological stages. According to the results of the GEPIA2 database, PLK4 was not significantly differentially expressed in different pathological stages of renal clear cell carcinoma in stages I, II, and III and slightly higher in stage IV (Figure 1(e)).

### 3.2. Micro-RNA Expression Analysis Date

To investigate the factors affecting the PLK4 expression, we used three databases, ENCORI, Target Scan, and TANRIC, to predict the micro-RNAs acting on target genes, and then used Veen plots to obtain an intersection of miRNA-has-miR-214-3p (Figure 2(a)), and we found that miRNA-has-miR-214-3p was highly expressed in normal tissues and lowly expressed in ccRCC (Figure 2(b)). The qPCR experiments showed that miRNA-has-miR-214-3p negatively regulated the expression of PLK4 (Figure 2(c)), while PLK4 was expressed at a higher level in ccRCC than in paracancerous tissues, suggesting that the high expression of PLK4 in ccRCC may be related to the low expression of miRNA-has-miR-214-3p in ccRCC.

### 3.3. Survival Prognosis Analysis Data

The results of the Kaplan-Meier plotter database survival analysis showed that high levels of PLK4 expression were an unfavorable prognostic factor for survival in patients with renal clear cell carcinoma (Figure 3(b)).

### 3.4. DNA Methylation of PLK4 and Its Prognostic Value in ccRCC

The DNA methylation level of PLK4 was significantly lower in ccRCC tumor tissues compared to paracancerous samples (Figure 4(a)). The methylation level of PLK4 was higher in high-grade tumors (Figure 4(b)) and advanced cancer stages (Figure 4(c)). In addition, after we analyzed the download methylation and gene expression raw dataset, the results showed that the PLK4 mRNA expression was significantly negatively correlated with its methylation status (Figure 4(d)). The predicted methylation sites of PLK4 showed three sites with high methylation levels in ccRCC include cg22112850, cg06015521, and cg26882168, of which the highest methylation level was found at cg22112850 (Figure 4(e)), indicating that the methylation level of PLK4 at this CpG site is mostly correlated with the prognosis of ccRCC (Table 1).

### 3.5. GO and KEGG Pathway Enrichment Analysis of PLK4-Related Gene

Based on the analysis results obtained by the STRING tool, we obtained a total of 17 PLK4 binding proteins (Figure 5(a)). We obtained 50 genes with similar functions to PLK4 from the GEPIA2 database and selected the top five genes with strong correlation for analysis. The results showed that the expression levels of PLK4 were positively correlated with the expression levels of KIF11, CCNA2, SKA3, CENPK, and BUB1B (Figures 5(b)–5(f)). GO analysis showed that PLK4 coexpressed genes are mainly involved in segregation, mitotic nuclear division, mitotic sister chromatid segregation, nuclear division, and organelle fission (Figure 5(g)). KEGG pathway analysis revealed that PLK4 was mainly enriched in the cell cycle, oocyte meiosis, progesterone-mediated oocyte maturation, cellular senescence, Hippo signaling pathway, human immunodeficiency virus 1 infection, circadian rhythm, homologous recombination, Fanconi anemia pathway, hedgehog signaling pathway, and P53 signaling pathway (Figure 5(h)).

### 3.6. PLK4 Is Correlated with Immune Infiltration in ccRCC

We used TIMER, CIBERSORT, TIDE, CIBERSORT-ABS, QUANTISEQ, XCELL, MCPCOUNTER, and EPIC algorithms to investigate the potential relationship between the level of infiltration of different immune cells and PLK4 gene expression in TCGA of different cancer types (algorithms were chosen based on all or most). The results showed that the PLK4 expression was positively correlated with the level of infiltration of cancer-associated fibroblast (rho = 0.269, *p* = 4.61*e* − 09), neutrophils (rho = 0.528, *p* = 1.86*e* − 34), myeloid dendritic cells (rho = 0.409, *p* = 5.33*e* − 20), active CD4^+^ T cells (rho = 0.292, *p* = 1.66*e* − 10), CD8^+^ T cells (rho = 0.358, *p* = 2.01*e* − 15), endothelial cells (rho = 0.166, *p* = 3.40*e* − 04), monocytes (rho = 0.418, *p* = 6.17*e* − 21), macrophage M1 (rho = 0.45, *p* = 2.60*e* − 24), and macrophage M2 (rho = −0.297, *p* = 8.10*e* − 11). Conversely, the PLK4 expression was correlated with the level of infiltration of NK cells (rho = −0.164, *p* = 4.00*e* − 04) (Figure 6(a)). In addition, PLK4 was significantly associated with genetic markers of neutrophils cells, dendritic cells, T cells, CD8^+^ T cells, TAM cells, monocyte cells, TAM cells, M1 macrophage cells, M2 macrophage cells, NK cells, Tfh cells, Treg cells, Th1 cells, Th2 cells, Th17 cells, and T cell exhaustion (Table 2). The PLK4 expression in ccRCC was significantly correlated with cytokines exerting immunosuppression, and most of them were positively correlated (Figure 6(b)), including CD96 (rho = 0.2952, *p* = 4.42*e* − 12), CD244 (rho = 0.2012, *p* = 3.15*e* − 06), CSF1R (rho = 0.231, *p* = 7.926*e* − 08), CTLA4 (rho = 0.2986, *p* = 2.456*e* − 12), IL10 (rho = 0.2717, *p* = 2.164*e* − 10), LAG3 (rho = 0.316, *p* = 1.046*e* − 13), LGALS9 (rho = 0.1896, *p* = 1.154*e* − 05), PDCD1 (rho = 0.2214, *p* = 2.745*e* − 07), PDCD1LG2 (rho = 0.3413, *p* = 7.154*e* − 16), TIGIT (rho = 0.3394, *p* = 1.069*e* − 15), and BTLA (rho = 0.321, *p* = 4.026*e* − 14) (Figure 6(c)). The immune cell phenotype (IPS) profile downloaded from TCIA was used to assess whether the PLK4 expression could predict the response to immunotherapy in ccRCC patients. IPS was significantly higher in the group with low PLK4 expression (Figure 6(d)), indicating that patients with lower PLK4 expression may have a better response to immunotherapy.

## 4. Discussion

PLK4 is involved in a variety of processes related to carcinogenesis, but it is unclear whether PLK4 is associated with the development and progression of ccRCC. This study is the first time to explore the expression, prognostic value, and potential effect on immune function of PLK4 in ccRCC through bioinformatics.

Based on the data analysis, we found that the expression level of PLK4 in ccRCC was significantly higher than that in the paracancerous tissue, i.e., PLK4 was highly expressed in ccRCC. The survival analysis of PLK4 using Kaplan-Meier plotter showed that the PLK4 expression was correlated with poor prognosis in ccRCC. Methylation and microRNA are two important means of affecting the gene expression [41]. Firstly, miRNA-has-miR-214-3p was predicated and experimentally verified to be a regulating miRNA of PLK4, which was found lowly expressed in ccRCC, but highly expressed in normal tissues from the GEO database. Obviously, the high expression of PLK4 in ccRCC may be associated with the miRNA-has-miR-214-3p low expression in ccRCC. To investigate the mechanism of PLK4 upregulation in more detail, the methylation levels of PLK4 in normal and cancerous tissues were analyzed using the UALCN database. The PLK4 mRNA expression was significantly negatively correlated with its methylation level, which was significantly lower in cancer tissues at various pathological stages and tumor grades, than in normal tissues. These results suggest that the high PLK4 expression in ccRCC may also be regulated by PLK4 methylation levels. In addition, the PLK4 methylation levels vary with ccRCC progression, indicating that PLKD methylation may also be a mechanism affecting ccRCC progression. To further pinpoint specific methylation sites, we used the MethSurv-A database to find the three sites with the highest methylation levels in PLK4, including cg22112850, cg06015521, and cg26882168, among which, the cg22112850 site had the highest methylation level, and analysis of its relationship with cancer prognosis revealed that the higher the methylation level of cg22112850 site, the better it was for cancer prognosis, and the cg22112850 site methylation might be beneficial for cancer prognosis. Therefore, the high expression of PLK4 in ccRCC may be mainly caused by the low expression level of miRNA-has-miR-214-3p and the low methylation level of PLK4 in ccRCC.

The abnormal proliferation of tumors and the formation of tumor immunosuppressive microenvironment provide the seeds and soil for tumor development, respectively [42, 43]. To understand the impact of PLK4 in aberrant tumor proliferation, we investigated and analyzed PLK4 coexpression genes to predict the role of PLK4 in aberrant tumor cell proliferation. PLK4 coexpressed genes are involved in and regulate the cell cycle, regulate centriole replication, and participate in cell mitosis. The expression of PLK4, an upstream regulator of centromeres, is closely related to centromere replication, and its abnormal expression can lead to an abnormal increase in the number of centromeres, causing centromere abnormalities, chromosome instability, and mitotic mutations [44]. It has been shown that the high PLK4 expression affects the cell cycle through the P38/P53/P21 signaling pathway, and inhibition of the PLK4 expression induces cell cycle arrest in the G1 phase [45]. By GO analysis, we found that PLK4 is closely related to the cell division process. During tumorigenesis and progression, PLK4 is overexpressed when the P53 signaling pathway is abnormal, leading to abnormal replication of centrioles, which in turn drives tumor development [46]. In our study, we found that PLK4 is associated with the P53 signaling pathway and affects the cell cycle. These results suggest that PLK4 has an important regulatory role in the process of cell division.

To understand the biological functions of PLK4 and the specific regulatory mechanisms and potential regulatory strategies in tumorigenesis and progression, we enriched the coexpressed genes of PLK4 and investigated its relationship with immune infiltration to explore the effects of PLK4 on the tumor cycle and the tumor microenvironment. Local infiltration of immune cells such as macrophages and T cells in the tumor is a major component of the tumor immune microenvironment [47, 48]. We found that the PLK4 expression was positively correlated with immune infiltration of most immune cells, including cancer-associated fibroblast, neutrophils, myeloid dendritic cells, active CD4^+^ T cells, CD8^+^ T cells, endothelial cells, monocytes, and macrophage M1, negatively correlated with NK cells and macrophage M2, and significantly correlated with genetic markers of CD8^+^ T cell, T cell, monocyte, TAM, M1 macrophage, M2 macrophage, neutrophils, NK cells, dendritic cells, Th1 cells, and Th2 cells. Macrophages mainly consist of macrophage M1 and macrophage M2. The M1 phenotype secretes proinflammatory cytokines and chemokines that cause inflammatory diseases and suppress tumorigenesis, while macrophage M2 promotes tumor development [49]. And CD8^+^ T cells, as immune surveillance cells, can inhibit tumor development by secreting cytokines to indirectly attack tumor cells [50, 51]. IPS data downloaded from TCIA provides predictive scores for assessing patient response to immunotherapy [52]. Our results showed higher IPS levels in the PLK4 low expression group, indicating that patients with the low PLK4 expression may have a better response to immunotherapy.

In addition, we further analyzed the correlation between the PLK4 expression and the expression of cytokines associated with exerting immunosuppression using the TISIDB database and showed that PLK4 expression levels also positively correlated with most of the cytokines exerting immunosuppression, including CD96, CD244, CSF1R, CTLA4, IL10, LAG3, LGALS9, PDCD1, PDCD1LG2, TIGIT, and BTLA. Although the infiltration of immune cells such as CD8^+^ T cells and macrophage M1 increased with the increase of PLK4 expression level, the expression level of PLK4 was also positively correlated with the tumor proliferation-promoting cytokines in the immunosuppressive microenvironment from the perspective of immunosuppressive cytokines; so, these cytokines may be involved in the formation of tumor immunosuppressive microenvironment.

## 5. Conclusion

In conclusion, our study identified the high PLK4 expression by bioinformatics analysis as a detrimental factor in the prognosis of ccRCC patients. The PLK4 expression may be negatively regulated by DNA methylation levels and miRNA expression and is associated with immune cell infiltration and exerting immunosuppressive cytokines; thus, PLK4 may be a potential target for clinical treatment of ccRCC.

## Figures and Tables

**Figure 1:** The high expression of PLK4 in ccRCC. (a) The expression of PLK4 in different human tumors from The Cancer Genome Atlas (TCGA) database was analyzed by the Tumor Immunity Estimation Resource (TIMER). PLK4 was upregulated in (b) analysis of PLK4 gene expression levels between ccRCC and its paraneoplastic tissues using the UALCAN database. (c) Differential expression of PLK4 in normal and cancerous tissues by the GEO database. (d) The differential expression of PLK4 in tumor tissues and their paired paracancerous tissues was obtained by paired sample analysis of TCGA. (e) The expression of PLK4 at different clinical stages in ccRCC. ^∗^*p* < 0.05, ^∗∗^*p* < 0.01, ^∗∗∗^*p* < 0.001.

**Figure 2:** The relationship between micro-RNA expression and PLK4 expression. (a) ENCORI, Target Scan, and TANRIC, three databases, predicted the role of PLK4 micro-RNA, and then the intersection was obtained with a Veen plot to get a miRNA-has-miR-214-3p. (b) The expression of miRNA-has-miR-214-3p in ccRCC and paraneoplastic samples. (c) Negative regulation of miR-214-3p and PLK4 expression as shown by qPCR. ^∗^*p* < 0.05; ^∗∗^*p* < 0.01; ^∗∗∗^*p* < 0.001; NS: not significant.

**Figure 3:** Effect of PLK4 on the survival prognosis of ccRCC patients. Kaplan-Meier survival analysis shows that high PLK4 expression is an unfavorable prognostic factor for survival in patients with ccRCC.

**Figure 4:** DNA methylation levels and sites of PLK4 and its effect on the prognosis of ccRCC. (a) Methylation levels of PLK4 in normal and ccRCC tissues by the UALCAN database. (b, c) Methylation levels of PLK4 in ccRCC tumor tissues of different tumor grades (b) and different tumor stages (c) by the UALCAN database. (d) Correlation analysis of PLK4 methylation levels in the cBioPortal database and RNA expression of PLK4 in UCSC website using *R* language. (e) Heat map of CpG sites for DNA methylation of PLK4 gene in the MethSurv database. ^∗^*p* < 0.05; ^∗^*p* < 0.01; ^∗∗∗^*p* < 0.001.

**Figure 5:** GO and KEGG pathway enrichment analysis of PLK4-related gene. (a) 17 binding proteins of PLK4 obtained were by the STRING database. (b)–(f) After the top 50 PLK4-related target genes were obtained from the GEPIA2 database, TIMER2 was applied to analyze the top 5 genes with strong PLK4 association. (g, h) The two sets of data were combined, and 64 genes were left after deleting duplicates for GO enrichment analysis (g) and KEGG pathway analysis with the *R* package, respectively (h).

**Figure 6:** (a)–(c) Correlation between PLK4 with immune infiltration in ccRCC. (a) Correlation between PLK4 expression and the abundance of tumor infiltrating immune cells in ccRCC available from the TIMER database. (b, c) Correlation between the PLK4 expression in ccRCC and cytokines exerting immunosuppression obtained from the TISIDB database (b), and the proteins that exert immunosuppression positively and strongly correlated with the PLK4 expression were plotted as scatter plots of their correlation in ccRCC (c). (d) The difference of IPS between the high- and low-PLK4 subgroups.^∗^*p* < 0.05; ^∗∗∗^*p* < 0.001; NS: not significant.

**Table 1:** The remarkable prognostic values of CpG in PLK4.

Gene symbol	Name	HR	CI	LR_test_pvalue	UCSC_RefGene_Group	Relation_to_UCSC_CpG_Island
PLK4	cg00608362	0.405	(0.226; 0.724)	0.00066^∗^	TSS200	Island
	cg02085815	0.387	(0.241; 0.621)	2.00*E*-05^∗∗∗^	TSS200	Island
	cg02994288	1.556	(1.054; 2.296)	0.025^∗^	TSS200	Island
	cg06015521	0.698	(0.472; 1.032)	0.072	Body	Open_Sea
	cg10393416	1.428	(0.858; 2.376)	0.15	1stExon; 5′UTR	Island
	cg11014917	0.674	(0.455; 0.998)	0.047^∗^	Body	Island
	cg17765713	1.411	(0.96; 2.076)	0.079	TSS1500	N_Shore
	cg20088535	0.55	(0.318; 0.951)	0.022^∗^	TSS200	Island
	cg21722058	0.545	(0.368; 0.807)	0.0022^∗∗^	1stExon; 5′UTR	Island
	cg22112850	0.684	(0.426; 1.097)	0.1	Body	S_Shelf
	cg23607253	0.611	(0.373; 1.001)	0.041^∗^	TSS200	Island
	cg23677608	0.492	(0.323; 0.75)	5.9*E*-04^∗∗∗^	TSS200	Island
	cg26882168	0.587	(0.385; 0.896)	0.018^∗^	3′UTR	Open_Sea

^∗^ *p* < 0.05; ^∗∗^*p* < 0.01; ^∗∗∗^*p* < 0.001.

**Table 2:** The correlation of PLK4 and immune cell gene markers in ccRCC by GEPIA.

Description	Gene markers	Purity cor.	*p* value
Neutrophils	CD66b (CEACAM8)	0.05	0.25
	CD11b (ITGAM)	0.059	0.18
	CCR7	0.099	2.30*E*-02^∗^

Dendritic cell	HLA-DPB1	0.16	1.90*E*-04^∗∗∗^
	HLA-DQB1	0.13	3.90*E*-03^∗∗^
	HLA-DRA	0.2	3.00*E*-06^∗∗∗^
	HLA-DPA1	0.19	1.10*E*-05^∗∗∗^
	BDCA-1 (CD1C)	0.065	0.14
	BDCA-4 (NRP1)	0.17	7.10*E*-05^∗∗∗^
	CD11c	0.2	2.60*E*-06^∗∗∗^

T cell (general)	CD3D	0.24	1.70*E*-08^∗∗∗^
	CD3E	0.26	9.40*E*-10^∗∗∗^
	CD2	0.32	2.90*E*-14^∗∗∗^

CD8+ T cell	CD8A	0.3	2.20*E*-12^∗∗∗^
	CD8B	0.24	2.70*E*-08^∗∗∗^

TAM	CCL2	-0.1	1.80*E*-02^∗^
	CD68	0.18	3.30*E*-05^∗∗∗^
	IL10	0.2	5.80*E*-06^∗∗∗^

Monocyte	CD86	0.31	2.20*E*-13^∗∗∗^
	CD115 (CSF1R)	0.26	1.10*E*-09^∗∗∗^

M1 macrophage	INOS (NOS2)	0.056	0.2
	IRF5	0.1	2.20*E*-02∗
	COX2 (PTGS2)	0.025	0.58

M2 macrophage	CD163	0.28	1.60*E*-10^∗∗∗^
	VSIG4	0.28	4.00*E*-11^∗∗∗^
	MS4A4A	0.27	5.20*E*-10^∗∗∗^

NK	KIR2DL1	-0.00032	0.99
	KIR2DL3	0.015	0.73
	KIR2DL4	0.12	6.70*E*-03^∗∗^
	KIR3DL1	-0.013	0.77
	KIR3DL2	0.027	0.54
	KIR3DL3	0.053	0.23
	KIR2DS4	0.033	0.45

Tfh	BCL6	0.16	1.50*E*-04^∗∗∗^
	IL21	0.27	5.20*E*-10^∗∗∗^

Treg	FOXP3	0.24	3.80*E*-08^∗∗∗^
	CCR8	0.3	4.00*E*-12^∗∗∗^
	STAT5B	0.13	3.50*E*-03^∗∗^
	TGF*β* (TGFB1)	0.31	3.10*E*-13^∗∗∗^

B cell	CD19	0.07	0.11
	CD79A	-0.007	0.87

Th1	T-bet (TBX21)	0.22	6.50*E*-07^∗∗∗^
	STAT4	0.24	4.90*E*-08^∗∗∗^
	STAT1	0.42	0
	IFN-*γ* (IFNG)	0.44	0
	TNF-*α* (TNF)	0.16	2.40*E*-04^∗∗∗^

Th2	GATA3	0.19	7.20*E*-06^∗∗∗^
	STAT6	0.15	6.40*E*-04^∗∗∗^
	STAT5A	0.26	2.80*E*-09^∗∗∗^
	IL13	0.027	0.54

Th17	STAT3	0.26	2.80*E*-19^∗∗∗^
	IL17A	-0.03	0.5

T cell exhaustion	PD-1 (PDCD1)	0.34	6.70*E*-16^∗∗∗^
	CTLA4	0.4	0
	LAG3	0.35	0
	TIM3 (HAVCR2)	0.016	0.72
	GZMB	0.33	4.00*E*-15^∗∗∗^

^∗^ *p* < 0.05; ^∗∗^*p* < 0.01; ^∗∗∗^*p* < 0.001.

## Data Availability

The gene expression profiling data supporting this study are from previously reported studies and datasets, which have been cited.
